# Regulation of Angiotensin- Converting Enzyme 2 in Obesity: Implications for COVID-19

**DOI:** 10.3389/fphys.2020.555039

**Published:** 2020-09-18

**Authors:** Saba Al Heialy, Mahmood Yaseen Hachim, Abiola Senok, Mellissa Gaudet, Ahmad Abou Tayoun, Rifat Hamoudi, Alawi Alsheikh-Ali, Qutayba Hamid

**Affiliations:** ^1^College of Medicine, Mohammed Bin Rashid University of Medicine and Health Sciences, Dubai, United Arab Emirates; ^2^Meakins-Christie Laboratories, Research Institute of the McGill University Health Center, Montreal, QC, Canada; ^3^Al Jalila Children’s Specialty Hospital, Dubai, United Arab Emirates; ^4^Sharjah Institute for Medical Research, College of Medicine, University of Sharjah, Sharjah, United Arab Emirates

**Keywords:** obesity, ACE2, COVID-19, SARS-CoV-2, lipid metabolism

## Abstract

The ongoing COVID-19 pandemic is caused by the novel coronavirus SARS-CoV-2. Age, smoking, obesity, and chronic diseases such as cardiovascular disease and diabetes have been described as risk factors for severe complications and mortality in COVID-19. Obesity and diabetes are usually associated with dysregulated lipid synthesis and clearance, which can initiate or aggravate pulmonary inflammation and injury. It has been shown that for viral entry into the host cell, SARS-CoV-2 utilizes the angiotensin-converting enzyme 2 (ACE2) receptors present on the cells. We aimed to characterize how SARS-CoV-2 dysregulates lipid metabolism pathways in the host and the effect of dysregulated lipogenesis on the regulation of ACE2, specifically in obesity. In our study, through the re-analysis of publicly available transcriptomic data, we first found that lung epithelial cells infected with SARS-CoV-2 showed upregulation of genes associated with lipid metabolism, including the *SOC3* gene, which is involved in the regulation of inflammation and inhibition of leptin signaling. This is of interest as viruses may hijack host lipid metabolism to allow the completion of their viral replication cycles. Furthermore, a dataset using a mouse model of diet-induced obesity showed a significant increase in *Ace2* expression in the lungs, which negatively correlated with the expression of genes that code for sterol response element-binding proteins 1 and 2 (SREBP). Suppression of *Srebp1* showed a significant increase in *Ace2* expression in the lung. Moreover, *ACE2* expression in human subcutaneous adipose tissue can be regulated through changes in diet. Validation of the *in silico* data revealed a higher expression of *ACE2, TMPRSS2* and *SREBP1 in vitro* in lung epithelial cells from obese subjects compared to non-obese subjects. To our knowledge this is the first study to show upregulation of ACE2 and TMPRSS2 in obesity. *In silico* and *in vitro* results suggest that the dysregulated lipogenesis and the subsequently high ACE2 expression in obese patients might be the mechanism underlying the increased risk for severe complications in those patients when infected by SARS-CoV-2.

## Introduction

As the COVID-19 pandemic continues, people worldwide are warned to take necessary precautions to avoid infection. With changing statistics every day, it is clear that certain groups of individuals are at increased risk of severe infection. In particular, the groups at risk are the elderly, individuals with chronic health conditions such as diabetes, cancer, and cardiovascular diseases. Most cases of COVID-19 are classified as mild or moderate. However, some cases are severe and may lead to acute respiratory distress syndrome (ARDS) and even death in those infected (Velavan and Meyer, 2020). Therefore, it is crucial to understand the mechanism by which this virus causes organ injury and, in particular, the immune system, which is mounted in response to the infection. A few studies have now identified other risk factors for severe complications and death due to COVID-19, namely smoking and obesity (Lighter et al., 2020; Patwardhan, 2020). The findings related to obesity are plausible since obese individuals tend to be more difficult to intubate, and excess body weight may contribute to increased pressure on the diaphragm, which may make breathing more difficult during infection. Moreover, it is well established that obesity leads to chronic meta-inflammation even in the absence of infection, which has detrimental effects on the immune system such as polarization of macrophages toward a pro-inflammatory phenotype termed M1 macrophages (Li et al., 2018). Other effects of obesity on the immune system include polarization of T cells toward a pro-inflammatory Th17 phenotype through the accumulation of dendritic cells in the adipose tissue (Woltman et al., 2007) and release of superoxide ion by neutrophils in the adipose tissue (Brotfain et al., 2015). In addition, obesity is associated with dysregulated lipid synthesis and clearance, which can initiate or aggravate pulmonary inflammation. It has also been shown that antiviral medication and vaccines are less effective in obese individuals (Painter et al., 2015). In relation to the influenza virus, obesity may have a role in the viral life cycle, which, along with a dysregulated immune system, could lead to severe complications (Honce and Schultz-Cherry, 2019). During the H1N1 pandemic in 2009, obesity was classified as an independent risk factor for hospitalization, need for mechanical ventilation, and death (Morgan et al., 2010). These observations are concerning since over one-third of the world population are classified as overweight or obese (Hruby and Hu, 2015). Therefore, in the ongoing COVID-19 pandemic, it is important to understand the molecular mechanisms through which obesity increases the complications related to COVID-19 to hopefully be able to design more appropriate therapies. Moreover, understanding the effects of obesity on COVID-19 may shed light on the pathogenicity of SARS-CoV-2.

The mode of cellular entry of the novel severe acute respiratory syndrome coronavirus, SARS-CoV-2, is through its binding to the angiotensin-converting enzyme 2 (ACE2) and is similar to SARS-CoV responsible for the 2003 pandemic (Lake, 2020). Specifically, the spike glycoprotein on the virion binds to the peptidase domain of ACE2. Moreover, it has been shown that the serine protease TMPRSS2 is used by SARS-CoV-2 for the S protein binding (Hoffmann et al., 2020). Physiologically, ACE2 is part of the renin-angiotensin system (RAS) and serves as a key regulator of systemic blood pressure through the cleavage of Angiotensin (Ang) I to generate the inactive Ang 1–9 peptide, and it directly metabolizes Ang II to generate Ang 1–7 limiting its effects on vasoconstriction and fibrosis. Other than serving as a functional receptor for SARS-CoV, ACE2 has been shown to be implicated in cardiovascular pathologies, diabetes, and lung disease. It is expressed by cells of the heart, kidney, and more specifically in lung epithelial cells (Oudit et al., 2009). Although ACE2 expression correlates with susceptibility of SARS-CoV infection, the relationship between ACE2 and SARS-CoV-2 is yet to be fully elucidated. In fact, studies have suggested a protective role for ACE2 where overexpression of ACE2 attenuates lung inflammation (Gu et al., 2016). Current research is focusing on the regulation and role of this receptor in relation to SARS-CoV-2. The aim of this study was to identify mechanisms, through re-analysis of publicly available transcriptomic data, by which SARS-CoV-2 dysregulates the lipid mechanism pathways and investigate the effect of dysregulated lipogenesis on the regulation of ACE2, specifically in obesity.

## Materials and Methods

### Differentially Expressed Genes in Bronchial Epithelial Cells Infected With SARS-CoV-2

In order to identify essential differentially expressed genes (DEGs) in SARS-CoV-2 infected versus non-infected epithelial cells, we re-analyzed the publicly available transcriptomic dataset (GSE147507) recently uploaded to the Gene Expression Omnibus (GEO) (Blanco-Melo et al., 2020). Independent biological triplicates of primary human lung epithelium (NHBE) were mock-treated or infected with SARS-CoV-2 (USA-WA1/2020), then subjected to whole transcriptomic analysis using RNA-Sequencing on Illumina Next Seq 500. The Raw Read Counts were retrieved and filtered from non-expressing genes that showed zero counts in the six samples. Out of the original 23,710 genes, only 15,487 were expressed and selected for further analysis. The filtered gene expression was uploaded to AltAnalyze software for Comprehensive Transcriptome Analysis (Emig et al., 2010). Principle component analysis and Heatmap clustering were generated, and DEGs were identified using LIMMA algorithm built-in AltAnalyze software. The genes that made the optimal hierarchal cosine clustering were identified, and the common pathways shared by these genes are listed according to their significance. Graphical visualization of the gene was made using the Metascape online tool for gene ontology^1^ (Zhou et al., 2019).

### Cell Culture

Normal human primary bronchial epithelial (NHBE) cells from non-obese (BMI < 30 kg/m^2^) and obese (BMI ≥ 30 kg/m^2^) subjects were purchased from a commercial source (MatTek, MA, United States) or obtained from the Biobank of the Quebec Respiratory Health Research Network at the Meakins-Christie Laboratories, Research Institute of the McGill University Health Centre. Table 1 shows the data from the non-obese and obese subjects. NHBE cells were cultured in BEGM media (Lonza, MD, United States) supplemented with 1% antibiotic antimycotic solution (Wisent, QC, Canada) in tissue culture flasks coated with Type 1 Rat tail collagen (Sigma-Aldrich, Ontario, ON, Canada). Cells were grown to 90% confluency and detached using 0.05% Trypsin-EDTA (Thermo Fisher Scientific, MA, United States). Fifty thousand cells were reserved for RNA extraction.

**TABLE 1:** Characteristics of non-obese and obese lung epithelial cells.

	**Non-obese**	**Obese**
N	4	3
Age, yr	42.3 ± 7.5	46.3 ± 6.1
BMI, kg/m2	23.6 ± 5.4	37.3 ± 3.1

*Values are mean ± SEM. BMI, body mass index.*

### RNA Extraction and Quantitative Reverse Transcription Polymerase Chain Reaction

Extraction of total RNA from NHBE cells was performed using a phenol-chloroform extraction (RiboZol RNA extraction reagent, VWR, Leicestershire, United Kingdom), as directed in the manufacturer’s instructions. Contaminating DNA was removed from 500 ng of total RNA using the AccuRT Genomic DNA Removal Kit (Applied Biological Materials, Richmond, BC, Canada), following manufacturer’s protocol. Reverse transcription was performed using the 5× All-In-One Reverse Transcriptase Mastermix (ABM). Expression of ACE2 mRNA and GAPDG (house keeping gene) were measured using EvaGreen qPCR Mastermix (ABM). Table 2 shows forward, and reverse primers used. The reaction was as follows: 5 μl of EvaGreen Mastermix, 2 μl of diluted cDNA (1/5), 0.6 μl of forward and reverse primers (10 μM) and 2.4 μl of nuclease free H_2_O. Each sample was tested in duplicates and the quantitative reverse transcription polymerase chain reaction (qPCR) amplification was performed using CFX96 thermal cycler (BioRad, Hercules, CA, United States) and cycler conditions were performed according to manufacturer’s protocol. The ΔΔCT method was used to measure gene expression: amount of target = 2^–ΔΔCT^.

**TABLE 2:** Forward and reverse primers of ACE2, TMPRSS22, SREBP1, and house keeping gene (GAPDH).

**Primer name**	**Oligo sequence (5′ to 3′)**
ACE2 forward	TCCATTGGTCTTCTGTCACCCG
ACE2 reverse	AGACCATCCACCTCCACTTCTC
TMPRSS2 forward	CCTCTAACTGGTGTGATGGCGT
TMPRSS2 reverse	TGCCAGGACTTCCTCTGAGATG
SREBP1 forward	ACTTCTGGAGGCATCGCAAGCA
SREBP1 reverse	AGGTTCCAGAGGAGGCTACAAG
GAPDH forward	GAAGGTGAAGGTCGGAGT
GAPDH reverse	GAAGATGGTGATGGGATTTC

## Results

### SARS-CoV-2 Differentially Expressed Genes Related to Lipid Metabolism in Epithelial Cells

A total of 121 DEGs in infected versus non-infected cells were identified, and they clustered the two groups separately (Figure 1). As expected, the top pathways where the DEGs by SARS-CoV-2 are involved were related to inflammatory, immune, cytokines, and antiviral responses.

**FIGURE 1:** Heatmap and clustering of SARS-CoV-2 infected healthy epithelial cells versus non-infected (mock-infected cells) using GSE147507 publicly available transcriptomics dataset. Pathways, where the DEGs are involved, are shown on the right side of the heatmap with their adjusted *p*-value. The C1 represent pathways of genes downregulated in infected cells, while C2 represent pathways of genes upregulated when cells are infected compared to mock-infected cells.

### Top DEGs in Infected Cells Can Have a Role in White Fat Differentiation

Of note, as shown in Figure 1, genes involved in lipid storage and high-density lipoprotein particles were among the top upregulated genes by the virus. To have a detailed analysis of the pathways where the top DEGs in infected versus non-infected epithelial cells are involved, we uploaded the 121 DEGs to metascape online tool. Again, most of the DEGs were involved in immune response-related such as Interleukin (IL)-17 signaling pathway. This result was expected and validated our bioinformatics analysis (Wu and Yang, 2020). IL-10 signaling pathway, acute inflammatory response, metal sequestration by antimicrobial proteins, defense response to another organism, negative regulation of apoptotic signaling pathway, acute-phase response, cellular response to tumor necrosis factor, response to antibiotic and modulation by a host of the viral process (Figure 2 and Table 3) were also involved. Other sets of enriched pathways are related to cell and tissue homeostasis like positive regulation of cell migration, blood vessel morphogenesis, regulation of bone resorption, activation of matrix metalloproteinases, and regulation of smooth muscle cell proliferation. The third set was related to metabolic pathways like negative regulation of ion transport, regulation of glucose metabolic process, the release of cytochrome c from mitochondria, and regulation of fat cell differentiation.

**FIGURE 2:** Heatmap of top Gene Ontology (GO) of the top DEGs in infected normal epithelium versus mock-infected cells. The bars represent the –log10 of the adjusted *p*-value for each pathway.

**TABLE 3:** Top Gene Ontology (GO) of the top DEGs in infected normal epithelium versus mock-infected cells and the symbols of genes in each pathway.

**Category**	**Term**	**Description**	**LogP**	**Log (*q*-value)**	**InTerm_InList**	**Symbols**
KEGG Pathway	hsa04657	IL-17 signaling pathway	–13.7848	-9.466	12/93	*CSF2, CSF3, CXCL3, IL6, CXCL8, MMP9, MMP13, S100A7, S100A8, CCL20, CXCL5, TNFAIP3, C3, CAMP, ICAM1, MAOB, IL36G, PGLYRP4, ZC3H12A, KLHL6, GSDMA, SSC5D, SERPINA3, LTB, MMP11, TNFSF14, SEMA3G, C1QTNF1, ADAM32, S100A7A, CSF1R, IFI6, IFI27, MX1, SAA1, SOD2, XAF1, CFB, C8B, SAA4, EGR2, ESRRB, PDK4*
Reactome gene sets	R-HSA-6783783	Interleukin-10 signaling	–7.09786	-3.779	6/47	*CSF2, CSF3, ICAM1, IL6, CXCL8, CCL20, LTB, CXCL5, C3, CXCL3, MMP9, SAA1, C8B, CAMP, TNFAIP3, EGR2, CSF1R, MX1*
GO biological processes	GO:0002526	Acute inflammatory response	–7.05687	-3.779	10/222	*SERPINA3, CFB, C3, C8B, ICAM1, IL6, S100A8, SAA1, SAA4, VNN1, MMP9, TNFAIP3, ZC3H12A, IL36G, CAMP, PGLYRP4*
Reactome gene sets	R-HSA-6799990	Metal sequestration by antimicrobial proteins	–5.71647	-2.740	3/6	*S100A7, S100A8, S100A7A, TNFAIP3, VNN1, CAMP, PGLYRP4, SERPINA3, C3, CSF2, IL6, CXCL8, MMP9, ZC3H12A, ICAM1, TCIM, SOD2, RNF183, IFI6*
GO biological processes	GO:0098542	Defense response to other organism	–5.39645	-2.446	13/596	*CAMP, IFI6, IFI27, IL6, MX1, S100A7, S100A8, CCL20, TNFAIP3, PGLYRP4, ZC3H12A, GSDMA, SSC5D*
GO biological processes	GO:0030335	Positive regulation of cell migration	–4.93817	-2.096	12/560	*CSF1R, ICAM1, IL6, CXCL8, MMP9, MYLK, S100A7, CCL20, SOD2, TNFSF14, SEMA3G, ZC3H12A, SAA1, C3, S100A8, C1QTNF1, MIR503*
GO biological processes	GO:2001234	Negative regulation of apoptotic signaling pathway	–4.87469	-2.047	8/233	*CSF2, IFI6, ICAM1, MMP9, SOD2, TNFAIP3, VNN1, PAK5, S100A8, RNF183, IFI27*
GO biological processes	GO:0048514	Blood vessel morphogenesis	–4.719	-1.931	13/690	*C3, IL6, CXCL8, MYLK, S100A7, TNFAIP2, TNFAIP3, FOXN1, KLF2, VASH1, ZC3H12A, THSD7A, MIR503, SOD2, MMP9, VNN1, C8B, ICAM1, KLHL6, SAA1, CSF1R, CSF2, LTB, SSC5D, C1QTNF1*
GO Biological processes	GO:0045124	Regulation of bone resorption	–4.3687	-1.652	4/42	*CSF1R, IL6, PDK4, TNFAIP3, SERPINA3, ESRRB, CSF2, CSF3, MMP9, ICAM1, FOXN1, VNN1, ZC3H12A, S100A8*
GO biological processes	GO:0006953	Acute-phase response	–4.17408	-1.492	4/47	*SERPINA3, IL6, SAA1, SAA4, CXCL8*
GO Biological Processes	GO:0071356	cellular response to tumor necrosis factor	–4.16725	-1.492	8/293	*ICAM1, CXCL8, LTB, CCL20, TNFAIP3, TNFSF14, KLF2, ZC3H12A, IL6, FOXN1*
GO biological processes	GO:0046677	Response to antibiotic	–3.8017	-1.253	8/331	*CSF3, ICAM1, IL6, MAOB, S100A8, TNFAIP3, KLF2, ZC3H12A, CXCL8, CCL20, CSF2, MMP9, SOD2, IFI6, PDK4, NID1, SAA1, TNFSF14, VNN1, C1QTNF1, MIR503, PFKFB1*
GO biological processes	GO:0044788	Modulation by host of viral process	–3.53447	-1.055	3/28	*CSF1R, IFI27, ZC3H12A, IFI6, MX1, XAF1, CAMP, PGLYRP4, IL6, TNFAIP3, CXCL8, ICAM1*
Reactome gene sets	R-HSA-1592389	Activation of matrix metalloproteinases	–3.32026	-0.899	3/33	*MMP9, MMP11, MMP13, IL6, ICAM1, NID1, COLGALT2, EGR2, PDK4, PFKFB1, TNFAIP3, KLF2, SERPINA3, ADAM32*
GO biological processes	GO:0043271	Negative regulation of ion transport	–3.01754	-0.715	5/162	*ICAM1, MAOB, MMP9, KCNE3, KCNRG, TNFAIP3, ZC3H12A, SSC5D*
GO biological processes	GO:0048660	Regulation of smooth muscle cell proliferation	–2.93566	-0.673	5/169	*IL6, MMP9, SOD2, TNFAIP3, MIR503*
GO biological processes	GO:0010906	Regulation of glucose metabolic process	–2.63653	-0.448	4/119	*ESRRB, PDK4, PFKFB1, C1QTNF1*
GO Biological processes	GO:0001836	Release of cytochrome c from mitochondria	–2.58309	-0.422	3/59	*IFI6, MMP9, SOD2, SERPINA3, C3, TNFSF14*
GO biological processes	GO:0045598	Regulation of fat cell differentiation	–2.40524	-0.306	4/138	*IL6, MMP11, ZC3H12A, PTPRQ, EGR2*
GO biological processes	GO:0001892	Embryonic placenta development	–2.05701	-0.084	3/91	*CSF2, ESRRB, VASH1*

*De novo* cellular lipogenesis, if disturbed, can change cell deformability as it influences the phospholipid composition of cellular membranes and, as a consequence, can disturb transmembrane receptors like growth factor receptor needed for cell survival (Stoiber et al., 2018). Based on that we were interested in deciphering the effect of viral infection on epithelial cells lipid metabolism pathways and how the disturbed lipid metabolism, like in obesity and diabetes, might worsen the condition of COVID-19.

### Negative Regulator of Lipogenesis Was Downregulated in Infected Cells

In this study, *IL6, MMP11, ZC3H12A, PTPRQ*, and *EGR2* were found to share a common pathway related to the regulation of fat cell differentiation. Of interest, *PTPRQ* and *EGR2* showed significant downregulation in infected cells compared to mock-infected epithelial cells, as shown in Figure 3. PTPRQ is protein tyrosine phosphatases (PTPs) that regulate tyrosine phosphorylation in signal transduction, and the encoded protein is a negative regulator of mesenchymal stem cell differentiation into adipocytes (Hale et al., 2017). It is synthesized in the lung and kidney and is downregulated in the early stages of adipogenesis (Thiriet, 2012). Recent studies linked downregulated PTPs like PTPRQ to lower weight gain, food intake, and leptin resistance (Shintani et al., 2017).

**FIGURE 3:** *PTPRQ* and *EGR2* are decreased in SARS-CoV-2 infected epithelial cells. Log10 of transcripts counts of the genes related to the regulation of fat cell differentiation IL6, MMP11, ZC3H12A, PTPRQ, and EGR2 in infected cells compared to mock-infected epithelial cells.

### SARS-CoV-2 Upregulate Leptin Signaling Regulator SOCS-3

Next, we tried to look for the trend of changes in the expression of genes involved in lipid metabolism (although the differences were not statistically significant), but this data can give us an idea about the deranged lipid-related pathways. To visualize the leptin signaling pathways, the filtered gene expression was uploaded to PathVisio pathway analysis and drawing software (Kutmon et al., 2015). As shown in Figure 4, there is derangement of a leptin signaling pathway in terms of upregulation or downregulation of genes involved, of note the *SOCS3, STAT1*, *NFKB1*, and *IL1B* were the top upregulated genes. Most individuals with obesity have leptin resistance by leptin and its receptor inhibitor *SOCS-3* (suppressor of cytokine signaling-3), leading to dysfunction of leptin biological function (Lubis et al., 2008).

**FIGURE 4:** Leptin signaling pathways genes members and their expression in SARS-CoV-2 infected epithelial cells versus non-infected. Red color signifies upregulation in infected cells, and green signifies downregulation as generated by PathVisio software.

### Lung ACE2 Expression Was Significantly Upregulated in Obese Mice

We then questioned whether disturbed lipid metabolism in obesity could affect the major players’ host genes involved in virus binding and entry, namely ACE2. Apart from the circulating RAS, the local lung-based RAS plays a specific role in the injury/repair response (Marshall, 2003) and recently was documented to have a pro-fibrotic effect independent of the known blood pressure effect (Wang J. et al., 2015). Recently, it was noted that COVID-19 can induce RAS imbalance that drives acute lung injury (Kickbusch and Leung, 2020). *In vitro* results showed that continued viral infection would reduce membrane ACE2 expression, leading to unstoppable activation of RAS in the lungs, which further induce local inflammation by recruited neutrophils after LPS stimuli (Vaduganathan et al., 2020). In COVID-19, ACE2 showed opposite harmful effects as an entry point, and beneficial effect by counteracting the overstimulated RAS as it degrades AngII to angiotensin 1–7 (Ang1–7) (Kuster et al., 2020). Interestingly Ang1–7 is shown to block high-fat diet-induced obesity, which increased ACE2 expression in adipose tissue (Patel et al., 2016). Therefore, our hypothesis was that induced obesity can upregulate ACE2 in the lung in response to a high-fat diet, which makes the lung more susceptible to viral entry but can regulate the overstimulated RAS. To examine that, we explored publicly available transcriptomics data, of studies where lungs were examined after inducing obesity, to look for the ACE2 expression changes. GSE38092 dataset was found with eight regular weight mice versus eight diet-induced obese mice where their lungs were extracted for microarray gene expression profiling (Tilton et al., 2013), as shown in Figure 5C. Interestingly, lung *Ace2* expression was significantly upregulated in obese mice compared to lean.

**FIGURE 5:** Ace2, *Srebf1*, and *Srebf2* expression are differentially expressed in obese mice. *Srebf1*, *Srebf2*, and *Ace2* mRNA normalized gene expression in response to a high-fat diet in obese compared to regular weight mice extracted from publicly available transcriptomic dataset GSE38092.

Sterol-response element-binding proteins (SREBP) are transcription factors that have been associated with lipogenesis, adipogenesis, and cholesterol homeostasis to prevent lipotoxicity. Studies have shown differential expression of SREBP-1 in regard to obesity. Figures 5A,B shows a decrease in *Srebf1* and *Srebf2*, the genes that code for the different proteins, namely SREBP-1 and SREBP-2.

The increased level of *Ace2* in the lungs of obese mice using publicly available datasets led us to investigate which cell type in the lung has the highest expression of *Ace2*. We explored LungGENS web-based tool that can map single-cell gene expression in the lung (Du et al., 2015). Among all cells in the human lungs, *Ace2* was expressed exclusively by epithelial cells, as shown in Figure 6.

**FIGURE 6:** Expression of ACE2 is highest in lung epithelial cells. mRNA expression of ACE2 was examined in different cell types within the lung using LungGENS web-based tool.

### Lung Epithelial Cells Express Lesser ACE2 During Activated Lipogenesis

The next question is how diet-induced obesity mechanistically can upregulate ACE2 in the lung, to answer this question, another dataset (GSE31797) was explored where the dynamics of lung lipotoxicity was examined by manipulating SREBP (Plantier et al., 2012). SREBPs regulate the expression of genes involved in lipid synthesis and function by their actions as transcription factors (Shimano and Sato, 2017). It was shown previously that the deletion of ACE2 in the liver and skeletal muscles could induce lipogenesis by inducing SREBPs, indicating the role of the ACE2/Ang1–7 axis in lipid metabolism (Cao et al., 2016, 2019).

In this dataset, alveolar type 2 cell RNA from Insig1/2Δ/Δ (activated SREBP1 levels) and Insig1flox/flox/Insig2−/− (suppressed SREBP1 levels) mice were profiled by microarray. Interestingly, activating SREBP1, coded by *Srebf1*, downregulated the expression of *Ace2* gene, as shown in Figure 7. This data indicates that *Ace2* expression might be under the control of SREBP1.

**FIGURE 7:** Ace2 expression is regulated by SREBP. Normalized mRNA expression of *Ace2* gene probes used in the publicly available dataset (GSE31797) comparing SREBP activated with SREBP inhibited alveolar cells.

### ACE2 Expression Is Regulated by Diet

In order to prove the effect of diet-induced changes in ACE2 expression, we used a publicly available subcutaneous adipose tissue transcriptomics dataset (GSE77962), where 25 males and 28 females (BMI = 28–35 kg/m^2^) followed a very-low-calorie diet (weight-loss period) for 5 weeks and a subsequent stable period for an additional 4 weeks (Johansson et al., 2012). Interestingly, we found in this dataset that there was a significant decrease in *ACE2* (*p* = 0.02) in individuals after weight loss compared to baseline (Figure 8). Moreover, this decrease was maintained when weight loss was stable. This data indicates a correlation between *ACE2* expression and diet.

**FIGURE 8:** *ACE2* expression is decreased in subcutaneous adipose tissue after weight loss. The following publicly available transcriptomic dataset (GSE77962) was explored (25 males; BMI: 28–35 kg/m^2^), and 28 females (BMI: 28–35 kg/m^2^) were placed on a very low-calorie diet for 5 weeks and a subsequent weight stable period for 4 weeks.

### qPCR Validation of *in silico* Analysis: ACE2 Expression Is Increased in Lung Epithelial Cells of Obese Subjects

Lung epithelial cells from non-obese and obese subjects were used to validate the *in silico* findings. Subjects selected had no other co-morbidities as to study the effect of obesity directly. Table 1 presents the data on the lung epithelial cells obtained from non-obese and obese subjects. ACE2 (*p* = 0.0005) and SREBP1 (*p* = 0.0015) expression were significantly increased in obese subjects as described in the *in silico* data (Figure 9). We were also interested to see the expression of TMPRSS2, a serine protease which is used by SARS-CoV-2 for S protein binding (Hoffmann et al., 2020). Following the trend of ACE2, TMPRSS2 was highly increase in obese lung epithelial cells as compared to lung epithelial cells obtained from non-obese subjects. To date, there are no *in vitro* studies on the expression of ACE2 in lung epithelial cells in the context of obesity.

**FIGURE 9:** ACE2, TMPRSS2, and SREBP1 expression are increased in lung epithelial cells of obese subjects. Lung epithelial cells from non-obese (*n* = 4) and obese (*n* = 3) were used to assess mRNA expression of ACE2 **(A)**, TMPRSS2 **(B)**, and SREBP1 **(C)**. **p < 0.01, ***p < 0.001.

## Discussion

This study, which uses publicly available data, demonstrates that SARS-CoV-2 infection induces changes in lipid profile in healthy hosts as demonstrated in infection of healthy epithelial cells. This is important when obesity is at play as the lipid profile is already disrupted, which may lead to increased susceptibility to infection which if occurs will further alter the lipid profile inducing hyper-inflammation.

Furthermore, our re-analysis of the publicly available transcriptomic datasets also demonstrated that SARS-CoV-2 infection of healthy epithelial cells compared to mock-infected cells clusters the genes involved in inflammatory, immune and viral responses (Figure 1). In particular, the IL-17 and IL-10 signaling pathways were heavily impacted. Symptoms of severe COVID-19 have been associated with a cytokine storm with high levels of IL-17, IL-10, IL-1β, IL-2, IL-7, IL-8, IL-9, among many other pro-inflammatory cytokines (Huang et al., 2020; Wu and Yang, 2020). IL-17, with its many pro-inflammatory effects, has been suggested as a potential target for the treatment of COVID-19. This is of interest as obesity is associated with high levels of immune cells producing IL-17 (Chehimi et al., 2017). IL-10, an anti-inflammatory cytokine with antiviral properties, is usually downregulated in infections. However, severe cases of COVID-19 have been associated with high levels of IL-10.

Obesity is a major health problem associated with an increased risk of developing diabetes, hypercholesteremia, and hypertension. Alterations in the metabolic pathways are seen, such as increases in leptin and insulin secretion and a decrease in adiponectin. Leptin stimulates fatty acid oxidation and may lead to lipotoxicity through decreased lipid accumulation in non-adipose tissue. As metabolic regulation and immune responses seem to be integrated with the function of one is dependent on the other, obesity is associated with high levels of pro-inflammatory mediators (Hotamisligil, 2006). Therefore, we focused our study on metabolic pathways in conjunction with inflammatory pathways. *In silico* analysis revealed that among the pathways that were differentially expressed were the regulation of glucose metabolic process and regulation of fat cell differentiation (Figure 2). *PTPRQ* and *EGR2* genes were significantly downregulated in SARS-CoV-2 infected healthy epithelial cells. Although they have been described to have roles in lipogenesis, their exact role in viral infection remains unknown and warrants further investigation.

The upregulation of *LEPR* and *LEP* and associated *SOC3* in response to SARS-CoV-2 infection was in line with mechanisms that are dysregulated in the state of obesity. This finding is of interest as it has been previously shown that viruses such as the West Nile Virus hijack cellular cholesterol to redistribute it and allow completion of its replication cycle (Mackenzie et al., 2007; Zhang et al., 2017). Previous studies have shown that obesity is associated with leptin resistance and increased blood levels of leptin with concomitant increases in *SOC3*, which plays a role in inhibiting signal transduction of leptin and other cytokines (Wunderlich et al., 2013).

Having established that SARS-CoV-2 infection and obesity share common pathways associated with dysregulation of lipid metabolism, we were interested to see if obesity, which has been described as a risk factor of COVID-19, is associated with higher susceptibility to infection. SARS-CoV-2 uses the ACE2 as a receptor for viral entry, so we hypothesized that obesity might lead to higher expression of ACE2. We first analyzed a dataset using a high-fat diet animal model of obesity, results revealed a higher expression of *Ace2* among diet-induced obese mice compared to lean mice. The data also suggests that ACE2 is largely expressed in epithelial cells of the lung. Previous studies with SARS-CoV have shown that the infection state correlates with the state of cell differentiation and expression of *ACE2* (Jia et al., 2005).

To validate these findings, lung epithelial cells were used from non-obese and obese subjects. To our knowledge, this is the first study to show that ACE2 and TMPRSS2, two entry points for SARS-CoV-2, are highly upregulated in lung epithelial cells from obese subjects using *in vitro* experiments.

The present study focused on the relationship between ACE2 expression and dysregulation of lipid metabolism. Therefore, we were interested to see how dysregulation of lipid metabolism could affect ACE2 expression. SREBPs are a family of transcription factors that control lipid synthesis and adipogenesis by controlling enzymes required for cholesterol, fatty acid, triacylglycerol, and phospholipid synthesis. In cholesterol deprivation, they translocate from the endoplasmic reticulum to the Golgi apparatus, where they are then targeted to the nucleus following cleavage. In the nucleus, they proceed to induce the expression of fatty acid and sterol synthesis (Bertolio et al., 2019). SREBP family is composed of SREBP-1 and SREBP-2. SREBP-1 exists as two isoforms: SREBP1-a and SREBP1-c. These isoforms are controlled by independent regulatory proteins and appear to respond differently to different states of lipid factors. *In silico* data suggests that suppressing SREBP1 leads to the upregulation of ACE2 expression. Of interest, analysis of another dataset revealed changes in ACE2 expression in adipose tissue of overweight or obese individuals who underwent a weight loss program. This result further emphasizes the relationship between ACE2 and weight and shows the modulation of ACE2 expression. De Macedo et al. (2015) showed that activation of ACE2 using diminazene aceturate had a significant effect on lipogenesis. *In vitro*, we found that SREBP1 expression is also upregulated in lung epithelial cells of obese subjects compared to non-obese subjects. In studies in chronic kidney disease it has been shown that angiotensin II activates SREBP1 which mediates angiotensin II–induced profibrogenic responses (Wang T.N. et al., 2015). In the present study, we have used a single cell model (lung epithelial cells) and it would be of future interest to study the effects of other factors such the role of immune cells in the regulation of these genes. Therefore, the relationship between ACE2 and SREBP1 remains to be fully understood and warrants further investigation.

## Conclusion

In summary, our findings from the publicly available transcriptomic data show that SARS-CoV-2 infection has significant effects on pathways involved in lipid metabolism. The proposed mechanism is illustrated in Figure 10. *In silico* and *in vitro* results suggest that ACE2 expression is increased in obese subjects which may be due to dysregulation in lipid metabolism. Increased ACE2 expression leads to an increase in the viral entry of SARS-CoV-2, which utilizes ACE2 as a receptor. Upon entry of the virus, dysregulation in lipid metabolism leads to an increase in SREBP, which subsequently leads to a decrease in ACE2. Inhibition of ACE2 activity results in increased lipotoxicity and inflammation. This mechanism demonstrates the dual function of ACE2 in viral infection. This is of importance as dysregulation of lipid metabolism is a feature of obesity, one of the risk factors of COVID-19. More importantly, our data reveal that this increased susceptibility may be due to an increase in ACE2 expression in the lung. These findings may potentially aide us in understanding the increased susceptibility in relation to other risk factors such as diabetes and hypercholesteremia.

**FIGURE 10:** Summary of the proposed mechanism of SARS-CoV-2 infection in obese individuals. (1) ACE2 expression is increased in obese subjects due to dysregulation in lipid metabolism. (2) Increased ACE2 expression leads to an increase in the viral entry of SARS-CoV-2, which utilizes ACE2 as a receptor. (3) Upon entry of the virus, dysregulation in lipid metabolism leads to an increase in SREBP, which subsequently leads to a decrease in ACE2 (4). (5, 6) Inhibition of ACE2 activity results in increased lipotoxicity and inflammation. This mechanism demonstrates the dual function of ACE2 in viral infection.

## Data Availability Statement

Publicly available datasets were analyzed in this study. This data can be found here: https://www.ncbi.nlm.nih.gov/geo; IDs: GSE147507, GSE38092, GSE31797, and GSE77962.

## Ethics Statement

Ethical review and approval was obtained from McGill University Health Centre Research Ethics Board (2021-6961). Written informed consent for participation was not required for this study in accordance with the national legislation and the institutional requirements.

## Author Contributions

SA, MH, AS, and MG designed the experiments, analyzed the samples, and contributed to data interpretation and manuscript preparation. AA, RH, AA-A, and QH contributed to data interpretation and manuscript preparation. All authors read and approved the final version of the manuscript.

## Conflict of Interest

The authors declare that the research was conducted in the absence of any commercial or financial relationships that could be construed as a potential conflict of interest.

## Footnotes

1 http://metascape.org
